# Study on the Mechanism and Oxidative Stress of Compound Danshen on the Degradation of Cx43 and Improvement of Myocardial Apoptosis in ICM Rats

This article has been retracted.

**DOI:** 10.1155/2022/6850425

**Published:** 2022-04-12

**Authors:** XingHua Chen, JiZhuo Zhang, Lu Han

**Affiliations:** ^1^Beijing ShijiTan Hospital, Capital Medical University, 100038 Beijing, China; ^2^Beijing Chaoyang Hospital, Capital Medical University, 100020 Beijing, China

## Abstract

In order to investigate the mechanism by which *Salvia miltiorrhiza* degrades connexin 43 (Cx43) and improves myocardial cell apoptosis and oxidative stress in rats with myocardial ischemia (ICM), male SD rats of pure grade are selected (32 rats), adaptively bred for 1 week, and then bred in SPF medium. They are randomly divided into a normal group, a model group, a low-dose Danshen group, and a high-dose group, with 8 rats in each group. HE staining and immunohistochemistry are performed. Serum samples are detected using kits according to instructions, including nitric oxide (NO) and endothelin-1 (ET-1); malondialdehyde (MDA), ELISA for superoxide dismutase (SOD), and vascular cell adhesion molecules (VCAM-1); western blot for detection of cardiac Cx43 protein expression; immunohistochemistry to detect Cx43 expression; and detection of myocardial ischemia. For ICM rats, the application of high-dose compound *Salvia miltiorrhiza* can effectively prevent the degradation of Cx43 protein, improve the apoptosis of myocardial cells in rats, and have a certain protective effect on ischemic myocardium in rats.

## 1. Introduction

Recent studies have shown that myocardial fibrosis is closely related to a variety of heart diseases, such as hypertension, myocardial infarction, and chronic myocardial ischemia [1]. During the development of myocardial disease, with the increase of myocardial collagen synthesis and the degree of fibrosis, myocardial interstitial edema may aggravate, resulting in decreased myocardial compliance and increased stiffness, thereby affecting myocardial systolic function and relaxation. Ischemic cardiomyopathy (ICM) is a disease caused by coronary atherosclerosis, which causes the imbalance of myocardial oxygen supply and oxygen demand, resulting in myocardial cell reduction, necrosis, and myocardial fibrosis and myocardial scarring. It is also known as myocardial infarction or myocardial fibrosis [2]. With the development of ICM, heart failure accounts for more than half of the causes of chronic heart failure (CHF). In recent years, the trend of these data has been increasing year by year [3]. From the perspective of the pathophysiological mechanism of ICM, it is mainly due to ventricular remodeling, including myocardial cell remodeling and interstitial myocardial remodeling. The process includes myocardial cell degeneration, necrosis, and apoptosis, as well as changes in the composition and quantity of extracellular matrix. The changes in ventricular morphology, structure, and function, which lead to changes in ventricular morphology, are an important mechanism for the progressive development of chronic ischemic myocardium into ICM and CHF [4].

Therefore, reducing apoptosis and preventing or reversing ventricular remodeling are important means to delay the onset of CHF, and myocardial fibrosis may cause serious damage to myocardial function, the risk of surgical treatment is significantly increased, causing patients to lose the opportunity for surgery, and clinical procedures such as cardiopulmonary bypass after cardiopulmonary bypass are more difficult, and the mortality rate is increased [5]. In recent years, many scholars have gradually turned to traditional Chinese medicine for the treatment of ICM, but there are relatively few studies, especially the research on dose control, and there is still a lack of effective research. Based on this, this paper starts with the mechanism of ICM and analyzes the effect of different doses of compound *Salvia miltiorrhiza* in ICM rats. The report is as follows.

## 2. The Proposed Model

32 male SD rats of pure grade with a body weight of 190–252 g, mean value of (231.25 ± 20.33) g, and an age of 8 weeks are selected. The animals are provided by Lyra Bio. Compound Danshen tablets, consisting of *Salvia miltiorrhiza* extract, *Panax notoginseng* powder, and borneol, were purchased from Guangzhou Baiyunshan Hutchison Whampoa Traditional Chinese Medicine Company (lot no. Z44023372); small animal fan, type SAR-830, was purchased from ITC, USA; optical microscope, MOS type, was purchased from Olympus, Japan; multifunctional image analysis system, Media Cyber model, was purchased from the United States; centrifuge, model LDZ5-2, was purchased from Beijing Centrifuge Factory; slicer, model Leica electronic scale, and model Metter all purchased from Swiss CNC; pipette, model Eppendorf, drying oven, and low-temperature refrigerator are purchased from Sanyo, Japan; water bath box and medical microwave are purchased from Aidi Instrument Factory.

### 2.1. Model Preparation

All animals are acclimatized for 1 week and then housed in SPF medium. They are randomly divided into a normal group, a model group, a low-dose group of Danshen, and a high-dose group, with 8 rats in each group.

A model of ischemic cardiomyopathy is prepared by ligation of the left anterior descending coronary artery [5–7]: first, the rat is anesthetized, intubated, and connected to a ventilator; with the intersection of the midline of the clavicle and the fourth rib as the center, the skin and muscle layer are incised along the midline of the clavicle, and the annular muscle layer is sutured with a purse-string suture [8, 9]. The fourth rib is cut off, the heart is pulled out of the thoracic cavity with a ring hook, and the left anterior descending coronary artery is ligated with No. 4/0 silk thread at 1.5 mm below the left atrial appendage, which are indicator of success [10–12]. The normal group is only threaded at the same site without ligation, and other operations are the same as those in the model group.

### 2.2. Grouping and Breeding of Animals

32 SD rats are adaptively housed for 1 week after purchase, and 8 rats are selected as the normal group according to the random number table method. The normal group is routinely fed 4 weeks after surgery, and from week 3 onwards, 1 ml/100 g saline is administered by gavage in the morning and evening.

Model group: in this group, a model is first created and routine feeding is performed for 1 month. After 3 weeks, 1 ml/100 g of saline is administered in the morning and evening. Dose groups: routine feeding is performed for 4 weeks after modeling and from the third week, Danshen 0.3 g (kg/d) and 0.6 g (kg/d) combination tablets are orally administered in the morning and evening.

### 2.3. Experimental Method

#### 2.3.1. Materials

In the third week of modeling, 2 rats in each group are randomly selected and sacrificed under anesthesia; myocardial tissue from the noninfarcted area of the rats under coronary artery ligation is collected, processed according to the experimental requirements, divided into several parts, each 100 mg, fixed with 4% paraformaldehyde, usually dehydrated, dipped in wax, embedded, and used for HE staining. Rats in other groups are sacrificed after 2 weeks of gavage; rats are routinely dehydrated, waxed, embedded, sliced, baked, dewaxed, and placed in water for immunohistochemical reaction.

#### 2.3.2. HE Staining

Sections are deparaffinized twice in xylene for 5 min each; 100%, 95%, 85%, and 70% alcohol are added over 3 min to each gradient; then, distilled water is transferred to hematoxylin for staining for 10 min; rinse with water for about 10 s to remove the excess staining solution on the incision; after rinsing with running water for 30 minutes, you can see that the core is blue; then, briefly rinse with distilled water; stain with 0.1% eosin for 5 minutes; use 70%, 85%, 95%, and 100% dehydrated alcohol, 2 minutes for each gradient. Installation and sealing: add an appropriate amount of neutral rubber and then seal with a coverslip.

#### 2.3.3. Immunohistochemical Reaction

Citrate repair: first, take the dewaxed and dehydrated sections and then drop the antigen retrieval solution into them. After completion, place them in a microwave oven for 10 minutes. After taking them out, wait for them to cool naturally, and then apply PBS to them. Ishing: the ishing time is controlled to 2∼3 min, and it is ished 3 times; then, take the wet box and place the slices; add endogenous peroxidase at a concentration of 3%, incubate it at room temperature, and apply PBS to it. Ishing: the ishing time is controlled to 2∼3 min, and it is ished 3 times. The blocking solution is normal goat serum; first put it at room temperature for 30∼40 min, shake off the excess liquid, and do not need to ish; add the primary antibody to the slice, put it in a 4°C environment to wait for overnight treatments with PBS, control the ishing time to 5∼6 min, ish 3 times, then put the secondary antibody IgG fermented bean curd, and place it at room temperature. In the environment, after 20 min, it is ished with PBS, the ishing time is controlled to 5∼6 min, and it is ished 3 times; finally, SA/HRP is dropped into the slice and it is placed at room temperature. After 20 min, it is ished with PBS, the ishing time is controlled to 5∼6 min, and it is ished 3 times; after the completion of the DAB color development, first set the ratio of DAB and distilled water to 1 : 1 drop, mix it well, add it to the sliced specimen, and ish it with water for 6 minutes; parallel counterstaining is performed with hematoxylin, and after drying, it is resin mounted and observed under a microscope.

### 2.4. Detection Method

#### 2.4.1. Serum Sample Detection

The rats are anesthetized with chloral hydrate, 4 ml of blood is collected from the abdominal aorta and centrifuged at 3000 rpm for 10 minutes, the upper serum is collected, and nitric oxide (NO), endothelial nitric oxide synthase (eNOS), and endothelin 1 (ET-1) levels are detected according to the kit instructions.

#### 2.4.2. ELISA Detection Method

On the 21st day after the experimental treatment, blood is collected from the rat heart, placed in an anticoagulation tube, and stored in a refrigerator at 4°C for 24 hours. Malondialdehyde (MDA), superoxide dismutase (SOD), and vascular cell adhesion molecule (VCAM-1) are detected with each index detection kit, respectively.

#### 2.4.3. Western Blot Detection of Cx43 Cardiac Protein Expression

First, use scissors to cut the tissue with a weight of about 50 mg. After cutting, place it in a tissue homogenizer and perform homogenization, centrifugation, and secondary antibody ishing operations on it. After the operation is completed, place it at room temperature. Incubate with shaking, and after ishing is complete, it will develop. The protein content of connexin 43 (Cx43) is represented by the gray value observation (the gray value of the protein band = the gray value of the background/(the gray value of the internal reference band−the gray value of the background)), and the calculation result is represented as mean and standard deviation.

#### 2.4.4. Immunohistochemical Detection of Cx43 Expression

SP immunohistochemical detection of Cx43: first, the distribution of Cx43 is observed by using a light microscope, and semiquantitative analysis is performed at the same time; if brown particles are found, it indicated that Cx43 is positive, and dark blue nuclei are counterstained with hematoxylin. Image Pro Plus 6.0 image analysis software analyzes the expression of Cx43, analyzes the integral optical density (IOD) of the positive expression sites, and divides the IOD by the area to obtain the intermediate density. The higher the positive expression per unit area, the larger the value.

First, Evans blue is injected into the rat heart. After the injection, the heart is quickly cut open and the tissue is frozen at −20°C. After freezing, it is sliced and incubated at 37°C. Simultaneous TTC staining was performed for 15 minutes. Observe the color of the area, where blue is normal tissue, light red is ischemic but not infarcted area, and white is ischemic infarcted area. After digital imaging, the area of each region is measured by an image analysis system to calculate the degree of myocardial ischemia. Myocardial ischemia rate = ischemic area/total area.

In this study, all the data are organized and a corresponding database is established for it, and all the databases are entered into SPSS 26.0 for neutral data processing, in which the measurement data are tested for normality, expressed as (*x* ± *s*). The multigroup test is F for normality between groups, and the Mann–Whitney *U* test is for nonnormality. The rate is expressed as %, and the test is *χ*^2^. When *P* < 0.05, the difference between the data is statistically significant.

## 3. The Experimental Result

### 3.1. Comparison of Serum NO, eNOS, and ET in Rats

Compared with the normal group, the NO and eNOS in the model group are significantly decreased and the ET is significantly increased (both *P* < 0.05). ET is significantly decreased and the NO and eNOS in the high-dose compound *Salvia miltiorrhiza* group are significantly higher than those in the low-dose group, and the ET is significantly lower than that in the low-dose group (both *P* < 0.05), as shown in Table 1.

### 3.2. Comparison of Serum MDA, SOD, and VCAM-1 Contents in Rats

The MDA and VCAM-1 in the model group are significantly higher than those in the normal group, and the SOD activity is significantly lower than that in the normal group (all *P* < 0.05). VCAM-1 is decreased, SOD activity is increased, and the MDA and VCAM-1 in the high-dose compound *Salvia* group are significantly lower than those in the low-dose group, and the SOD activity is significantly higher than that in the low-dose group (all *P* < 0.05), as shown in Table 2.

### 3.3. Comparison of Cx43 Protein Levels in Rat Myocardium

Compared with the normal group, the Cx43 protein level in the model group is significantly decreased (all *P* < 0.05); while compared with the model group, the Cx43 protein level in the low-dose and high-dose groups of compound Danshen increased, and the high-dose compound Danshen increased. The Cx43 protein level in the group is significantly higher than that in the low-dose group (both *P* < 0.05), as shown in Table 3.  Figure 1 shows comparison of myocardial Cx43 protein levels of rats.

### 3.4. Comparison of Cx43 Expression in Rat Myocardium

As shown in Figure 2, after immunohistochemical reaction, Cx43 protein is mainly presented and localized in the cytoplasm and cell membrane. The color is mainly brown, and the expression is positive. The strong positive expression is dark brown particles, and the weak positive expression is light brown particles. Dark blue parts are the color of nuclei after hematoxylin counterstaining.  Figure 2(a) shows the strong positive expression of Cx43 protein in normal rat cardiomyocytes, and the distribution rule is as follows: it is located at the junction of the outer end of the myocytes, and a small amount is expressed on the side of the cell membrane, with a ladder-like distribution.  Figure 2(b) shows the positive expression of Cx43 protein in the model group; the distribution law is mainly as follows: the distribution of dark brown particles is relatively scattered and sparse, the connection between each outer end increases, and some positions are distributed on the side.  Figure 2(c) shows the weakly positive expression of Cx43 protein in the low-dose compound *Salvia* group rats; the distribution law is mainly as follows: there are more light brown particles and brown particles. Compared with the model group, the connection parts between the outer ends are gradually increased, and some are distributed at the lateral end connection.  Figure 2(d) shows the positive expression of Cx43 protein in the compound Danshen high-dose group of rats; the distribution law is mainly as follows: dark brown particles gradually increased, especially in the low-dose group and model group (both *P* < 0.05), other distributions are like the low-dose group.  Figure 3 shows statistical chart of Cx43 distribution in each group of rats.

### 3.5. Comparison of Measurement Results of Myocardial Ischemia Range in Rats

Compared with the normal group, the myocardial ischemia rate in the model group is significantly increased (all *P* < 0.05); while compared with the model group, the myocardial ischemia rate in the low-dose and high-dose compound Danshen groups decreased significantly. The myocardial ischemia rate in the high-dose *Salvia miltiorrhiza* group is significantly lower than that in the low-dose group (all *P* < 0.05), as shown in Table 4.

## 4. Result Analysis and Discussion

Ischemic cardiomyopathy, with heart failure due to myocardial fibrosis, is the terminal stage of various heart diseases. The 5-year survival rate of patients with clinical symptoms is similar to that of malignant tumors. The basic mechanism leading to the development of heart failure is myocardial remodeling. The excitability of angiotensin-aldosterone system is increased, and endogenous neuroendocrine factors are activated to promote myocardial remodeling. Therefore, blocking myocardial remodeling is the key to the treatment of heart failure. At present, diuretics, angiotensin-converting enzyme inhibitors (ACEI) or angiotensin receptor antagonists, and JB-receptor blockers have been listed as the basic treatment for heart failure, and the emergence of advanced heart failure that will delay patients receiving the timing of coronary artery bypass grafting has a serious impact on the duration of cardiac function recovery in perioperative patients. Therefore, whether traditional Chinese medicine treatment methods can be applied clinically to improve the cardiac function of such patients, improve the prognosis, and strive for the opportunity for surgery for some patients can provide a certain basis for clinical practice through experimental research.

When myocardial ischemia or blood oxygen occurs in the body, the function of the oxygen free radical scavenging system of myocardial cells will decrease, or even lose its function. At this time, the activity of the generating system will be significantly enhanced, and the generating system will reduce the oxygen free radicals. A large amount of release, far exceeding the scavenging ability of antioxidant enzymes, causes many metabolites to accumulate around cardiomyocytes, destroying the function and structural changes of cardiomyocytes, increasing cardiomyocyte apoptosis and myocardial tissue necrosis. In this study, NO and eNOS in the model group are significantly decreased and ET and myocardial ischemia rates are significantly increased (both *P* < 0.05), while the low-dose and high-dose compound Danshen groups significantly increased NO and eNOS in the rat model group. The ET and myocardial ischemia rates are significantly decreased, the NO and eNOS in the high-dose compound Danshen group are significantly higher than those in the low-dose group, and the ET and myocardial ischemia rates are significantly lower than those in the low-dose group (both *P* < 0.05). The improvement of myocardial ischemia in rats is better, and it also suggests that it plays a major role in the diseases caused by myocardial ischemia. Its components are compatible with *Panax notoginseng*, which can play a synergistic effect together to expand coronary arteries and enhance serum model. The levels of NO and eNOS in the group can reduce the levels of ET and myocardial ischemia, and at the same time, the area of myocardial ischemia can be reduced, which provides data support for the treatment of the clinical coronary ligation myocardial ischemia rat model.

Compound Danshen is a kind of drug with high effect of promoting blood circulation and removing blood stasis, and the effect of high dose is significantly better than that of low dose. Its main function is to nourish blood, soothe the nerves, and reduce swelling. In addition, Danshensu can improve vascular calcification in the body and also has anti-inflammatory, antiatherosclerotic, and antioxidant effects. Also, *Panax notoginseng* is warm in nature, belongs to the liver and stomach meridian, stops bleeding, disperses blood stasis, and relieves pain. In the Compendium of Materia Medica Supplements, there are relevant records that *Panax notoginseng* and ginseng are equally precious and can directly expand coronary blood vessels and improve myocardial hypoxia; the active ingredients of *Panax notoginseng* include *Panax notoginseng* saponins and amino acids, of which three hepta saponins have the effect of promoting blood circulation, and the application of large doses of *Panax notoginseng* also has the effect of promoting blood circulation. Studies have found that *Panax notoginseng* saponins can reduce serum creatine phosphokinase isoenzymes and ventricular premature beats in rats and have antimyocardial ischemia and antiarrhythmic effects. As an auxiliary prescription drug, it is recorded in the Romance of Cao: when you are alone, you are weak, and there are messengers who have merit. Modern research has found that borneol has anti-inflammatory and analgesic effects, reduces ischemic myocardial damage, and improves the bioavailability of other drugs. Borneol can double the biological activity of nitric oxide in the body and is often used clinically in the treatment of cardiovascular and cerebrovascular diseases. This study found that compared with the normal group, MDA and VCAM-1 in the model group are significantly increased and SOD activity and Cx43 protein level are significantly decreased (both *P* < 0.05); MDA and VCAM-1 are decreased, SOD activity and Cx43 protein level are increased, and MDA and VCAM-1 in the high-dose compound Danshen group are significantly lower than those in low-dose groupoid activity, and Cx43 protein level is significantly higher than that in the low-dose group (all *P* < 0.05); *in vivo*, SOD is an important enzyme for scavenging oxygen free radicals, and after the free radicals undergo chain and peroxidation reactions, the product is MDA. Both levels can show myocardial antioxidant capacity. VCAM-1 is an important adhesion factor, and its main role is to participate in the regulation of the body. When the body is in myocardial ischemia, many centrocytes will continue to accumulate in the center of the damaged cardiomyocytes, causing damage to the microcirculation of the body tissue. At the same time, many oxygen free radicals, peroxidase, and other related mediators can be released, which can aggravate myocardial tissue or cell damage.

## 5. Conclusion

During the pathogenesis of myocardial ischemia, Cx43 is a structural protein that is easily degraded. If the expression of this protein decreases, it can be rapidly dephosphorylated, and at the same time, the structure of the connexin will be remodeled, resulting in a decrease in the coupling between cells. This process is the basis of arrhythmia during myocardial ischemia. The scholar believes that when myocardial ischemia occurs in the body, oxidative stress may participate in the dephosphorylation of myocardial Cx43 cells, resulting in the occurrence of arrhythmia. Therefore, Cx43 protein is closely related to MDA and SOD. There is a significant correlation between the expression of VACM-1 and VCAM-1. By inhibiting the expression of VACM-1, the release of active substances such as oxygen free radicals and peroxidase can be reduced, and the degradation of Cx43 protein can be inhibited, which can protect cardiomyocytes. Although this study has achieved certain results, there are still some shortcomings. The compound Danshen has not been compared with other drugs. Therefore, in the future research, the application effect in myocardial ischemia compared with other drugs is aimed at clinical myocardial ischemia. The paper provides data support for treatment and prevention.

To sum up, the application of 0.6 g/kg/d high-dose compound Danshen tablets to ICM rats can effectively prevent the degradation of Cx43 protein, improve the apoptosis of myocardial cells in rats, and play a certain protective effect on ischemic myocardium in rats.

## Figures and Tables

**Figure 1:** Comparison of myocardial Cx43 protein levels of rats.

**Figure 2:** The expression of Cx43 in the myocardium of rats in each group (immunohistochemistry ×400): (a) the normal group; (b) the model group; (c) the low-dose group; (d) the high-dose group.

**Figure 3:** Statistical chart of Cx43 distribution in each group of rats (immunohistochemistry). Note: ^*∗*^ means compared with the normal group, △ means compared with the model group, and ▲ means compared with the low-dose group; *P* < 0.05.

**Table 1:** Comparison of serum NO, eNOS, and ET of rats ($\bar{x}$ ± *s*).

Group	NO	eNOS	ET
Normal	32.56 ± 6.85	66.81 ± 9.62	35.15 ± 8.75
Model	12.56 ± 2.73^*∗*^	34.15 ± 5.34^*∗*^	92.43 ± 20.12^*∗*^
Low dose	18.96 ± 4.39^*∗*^^△^	46.33 ± 7.28^*∗*^^△^	77.58 ± 15.62^*∗*^^△^
High dose	24.33 ± 5.18^*∗*^^△▲^	53.25 ± 8.46^*∗*^^△▲^	55.85 ± 12.86^*∗*^^△▲^
*F*	7.851	10.256	16.852
*P*	<0.001	<0.001	<0.001

^*∗*^ means compared with the normal group, △ means compared with the model group, and ▲ means compared with the low-dose group; *P* < 0.05.

**Table 2:** Comparison of serum levels of MDA, SOD, and VCAM-1 in rats ($\bar{x}$ ± *s*).

Group	MDA (nmol/ml)	SOD (U/ml)	VCAM-1 (pg/ml)
Normal	0.15 ± 0.02	86.15 ± 4.26	19.26 ± 3.26
Model	0.21 ± 0.06^*∗*^	65.58 ± 1.26^*∗*^	75.18 ± 13.15^*∗*^
Low dose	0.18 ± 0.04^*∗*^^△^	72.56 ± 2.13^*∗*^^△^	53.81 ± 6.25^*∗*^^△^
High dose	0.16 ± 0.03^*∗*^^△▲^	81.59 ± 3.23^*∗*^^△▲^	42.19 ± 5.49^*∗*^^△▲^
*F*	8.898	8.725	11.625
*P*	<0.001	<0.001	<0.001

^*∗*^ means compared with the normal group, △ means compared with the model group, and ▲ means compared with the low-dose group; *P* < 0.05.

**Table 3:** Comparison of Cx43 protein levels in rat myocardium ($\bar{x}$ ± *s*).

Group	*n*	Cx43
Normal	8	133.56 ± 25.89
Model	8	37.18 ± 12.17^*∗*^
Low dose	8	61.84 ± 8.23^*∗*^^△^
High dose	8	79.91 ± 9.89^*∗*^^△▲^
*F*		15.629
*P*		<0.001

^*∗*^ means compared with the normal group, △ means compared with the model group, and ▲ means compared with the low-dose group; *P* < 0.05.

**Table 4:** Comparison of the measurement results of myocardial ischemia range in rats.

Group	Myocardial ischemia rate (%)
Normal	0.00 ± 0.00
Model	14.58 ± 3.75^*∗*^
Low dose	9.62 ± 2.61^*∗*^^△^
High dose	6.71 ± 2.05^*∗*^^△▲^
*F*	13.526
*P*	<0.001

^*∗*^ means compared with the normal group, △ means compared with the model group, and ▲ means compared with the low-dose group; *P* < 0.05.

## Data Availability

The simulation experiment data used to support the findings of this study are available from the corresponding author upon request.

## References

[1] Li J., Wang D., Yi L. (2020). Daphnetin inhibits the c-Jun N-terminal kinase/nuclear factor*κ*B(JNK/NF-*κ*B)pathway and alleviates myocardial ischemia injury in rats. *Cell and Molecular Immunology Journal*.

[2] Gharishvandi F., Shafaroodi H., Mohammad Jafari R., Abdollahi A., Pasalar P., Dehpour A. R. (2022). The protective effect of *α*7‐nACh receptor and its interaction with 5‐HT1B/1D receptors in acute intestinal ischemia‐reperfusion injury in rats. *Fundamental & Clinical Pharmacology*.

[3] Stener-Victorin E., Waldenström U., Tägnfors U., Lundeberg T., Lindstedt G., Janson P. O. (2000). Effects of electro-acupuncture on anovulation in women with polycystic ovary syndrome. *Acta Obstetricia et Gynecologica Scandinavica*.

[4] Hong C., Xing-Yuan W., Bao-Ya Z. (2018). Clinica l experience in treating 78 cases of upper limb edema after breast cancer operation by WenYang HuoXue Ishing Prescription. *TMR Modern Herbal Med*.

[5] Chen W. R., Hu S. Y., Chen Y. D. (2015). Effects of liraglutide on left ventricular function in patients with ST-segment elevation myocardial infarction undergoing primary percutaneous coronary intervention. *American Heart Journal*.

[6] Liang P., Mao L., Ma Y. (2021). A systematic review on Zhilong Huoxue Tongyu capsule in treating cardiovascular and cerebrovascular diseases: pharmacological actions, molecular mechanisms and clinical outcomes. *Journal of Ethnopharmacology*.

[7] Ding W., Ji Q., Wei Q., Shi Y., Ma R., Wang C. (2015). Prophylactic application of an intra-aortic balloon pump in high-risk patients undergoing off-pump coronary artery bypass grafting. *Cardiology*.

[8] Zhang Z., Cui F., Cao C., Wang Q., Zou Q. (2022). Single-cell RNA analysis reveals the potential risk of organ-specific cell types vulnerable to SARS-CoV-2 infections. *Computers in Biology and Medicine*.

[9] Yang Y., Sun F., Chen H. (2021). Postnatal exposure to DINP was associated with greater alterations of lipidomic markers for hepatic steatosis than DEHP in postweaning mice. *The Science of the Total Environment*.

[10] Zou Q., Xing P., Wei L., Liu B. (2019). Gene2vec: gene subsequence embedding for prediction of mammalian N6-methyladenosine sites from mRNA. *RNA*.

[11] Chen J., Zou Q., Li J. (2022). DeepM6ASeq-EL: prediction of human N6-methyladenosine (m6A) sites with LSTM and ensemble learning. *Frontiers of Computer Science*.

[12] Zong X., Xiao X., Shen B. (2021). The N 6-methyladenosine RNA-binding protein YTHDF1 modulates the translation of TRAF6 to mediate the intestinal immune response. *Nucleic Acids Research*.

